The article "Human Epididymis Protein-4 (HE-4): A Novel Cross-Class Protease Inhibitor" was retracted in 2024. Reasons: duplicated images; overlap with earlier publications; unreliable data; concerns about the images.

# Human Epididymis Protein-4 (HE-4): A Novel Cross-Class Protease Inhibitor

**DOI:** 10.1371/journal.pone.0047672

**Published:** 2012-11-05

**Authors:** Nirmal Chhikara, Mayank Saraswat, Anil Kumar Tomar, Sharmistha Dey, Sarman Singh, Savita Yadav

**Affiliations:** 1 Department of Biophysics, All India Institute of Medical Sciences, New Delhi, India; 2 Department of Lab Medicine, All India Institute of Medical Sciences, New Delhi, India; New York University, United States of America

## Abstract

Epididymal proteins represent the factors necessary for maturation of sperm and play a crucial role in sperm maturation. HE-4, an epididymal protein, is a member of whey acidic protein four-disulfide core (WFDC) family with no known function. A WFDC protein has a conserved WFDC domain of 50 amino acids with eight conserved cystine residue. HE-4 is a 124 amino acid long polypeptide with two WFDC domains. Here, we show that HE-4 is secreted in the human seminal fluid as a disulfide-bonded homo-trimer and is a cross-class protease inhibitor inhibits some of the serine, aspartyl and cysteine proteases tested using hemoglobin as a substrate. Using SPR we have also observed that HE-4 shows a significant binding with all these proteases. Disulfide linkages are essential for this activity. Moreover, HE-4 is N-glycosylated and highly stable on a wide range of pH and temperature. Taken together this suggests that HE-4 is a cross-class protease inhibitor which might confer protection against microbial virulence factors of proteolytic nature.

## Introduction

Human and chimpanzee genomes are similar to the extent of nearly 90% but, there are differences which impart uniqueness to the human species as well as chimpanzees and reveal the intrinsic genetic differences in the expressions of genes. A sudden or adaptive evolution in some of the genes or genomic regions might be playing some essential part in these differences. Recent comparative analysis of human and chimpanzee genome sequences identified some 16 regions with high density of rapidly evolving genes [1]. One such region contains genes encoding whey acidic protein (WAP) domain proteins. This region on human chromosome 20q13 is called WAP four-disulfide core domain (WFDC) locus containing 14 genes encoding WFDC type proteinase inhibitors [2]. Apart from these 14 genes from the same locus there are at least four other proteins having WFDC domain but are present at different chromosomes (Ch. 16, 17 and X chromosome) [3]–[6] Amplification of the 20q12–13 region has been documented in breast and ovarian carcinoma [7]–[8]. Consistent with these studies, SLPI and elafin are known to be expressed in various carcinomas and implicated in initiation or progression of tumorigenesis [9]–[13].

The article "Human Epididymis Protein-4 (HE-4): A Novel Cross-Class Protease Inhibitor" was retracted in 2024. Reasons: duplicated images; overlap with earlier publications; unreliable data; concerns about the images.

Most of the members of the family with the exception of SLPI, elafin, KAL1, EPPIN and ps20 have not been examined at the protein level. SLPI, elafin and ps20, have been reported to be expressed in different cell types including airway epithelium and mucosal secretions from tissues including male reproductive tract, respiratory tract as well as in inflammatory cells like T-cells and macrophages [14]–[16]. Two types of functions attributed to this family of proteins are regulation of proinflammatory mediators and anti-bacterial or anti-fungal activity [17]–[18]. Anti-infective activity of SLPI, elafin, and pro-infection attributes of ps20 regarding HIV have also been uncovered [19].

Another member of the family, WFDC-2 or HE-4 (human epididymis protein-4) was found to be the most frequently upregulated in ovarian carcinomas [20]. This protein is also known as Epididymal secretory protein E4, Major epididymis-specific protein E4 and putative protease inhibitor WAP5. WFDC-2 gene product was originally thought to be a protein specifically expressed in the epididymis and was dubbed as a tissue marker for the same [21]. Later, it was found to be expressed in the oral cavity, respiratory tract, female genital tract and distal renal tubules. Evidence of its expression in the colonic mucosa has also been found [22]. Evidence of HE-4 expression in various tumor types of the lung including lung adenocarcinoma has also been reported [16]. HE-4 levels in the serum have been suggested to be a sensitive marker for ovarian cancer and protein used as a histological marker for ovarian cancer [23]–[25].

On the basis of structural and sequential similarity of HE-4 with other WAP proteins like SLPI and elafin it was suggested that the protein might have antiprotease activity within the male reproductive, oral and respiratory tract. Other than this suggestion of HE-4 working as an antiprotease, no work has been done to elucidate the role and/or structure of the protein. Even this claim projecting it as a protease inhibitor has never been tested. It seems plausible that HE-4 will have as yet undetermined pivotal roles in human physiology. An investigation of this demand detailed studies at the protein level. A prerequisite for the above said objective is a rapid and efficient method to generate sufficient amounts of protein. This paper reports an accessible and efficient purification of HE-4 protein from human seminal fluid. We have further characterized HE-4, and found it to be a cross-class protease inhibitor and show a significant binding with all the proteases tested.

## Results

### HE-4 purified from seminal fluid exists as a trimer

HE-4 was purified from normozoospermic pooled human seminal plasma. Heparin-sepharose unbound fraction was further fractionated on DEAE-sephacel. Seminal plasma fractionated into four main peaks on DEAE-sephacel (Fig. 1 A, B). All the peaks were further fractionated by sephadex G-75 size exclusion chromatography (data shown only for peak I of DEAE) and HE-4 immnuoreactivity was found in peak III of G-75 fractionation (Fig. 1E, lane II). Western blot of purified protein and whole seminal plasma showed a band of approximately 14 kDa (Fig. 1E) which was confirmed by SDS-PAGE of the same in reducing conditions (Fig. 1D lane III). Under non-reducing conditions, HE-4 was found to migrate as a single band of approximately 42 kDa (Fig. 1D lane II). This suggests that HE-4 exists as a disulphide bonded trimer in human seminal plasma and disulfide bond reduction provide a monomer of 14 kDa. Identity of HE-4 was also confirmed by LC-MS/MS (Table 1). Mascot score of identification for HE-4 was 123 and four peptides were matched. One previous study has reported HE-4 to be N-glycosylated in saliva [26]. We analyzed the glycosylation of HE-4 with PAS staining method (Fig. 2A). We treated HE-4 with PNGase F under denaturing conditions and compared it with the native protein. An approximate shift of 2.5 kDa in the migration of deglycosylated HE-4 in SDS-PAGE was observed compared to native protein (Fig. 2B). This confirmed that HE-4 in seminal fluid is N-glycosylated.

The article "Human Epididymis Protein-4 (HE-4): A Novel Cross-Class Protease Inhibitor" was retracted in 2024. Reasons: duplicated images; overlap with earlier publications; unreliable data; concerns about the images.

**Figure 1:** Purification of HE-4 protein from human seminal plasma using affinity, ion exchange and gel filtration chromatography. (**A**) Elution profile of anion exchanger DEAE sephacel. The peaks formed as a function of X-axis as elution volume in ml and Y-axis is mA at 280 nm. The second (….) line represents the gradient of NaCl. The first peak with black base given is the one where we found HE-4. (**B**) 12.5% SDS-PAGE of peaks obtained from anion exchanger DEAE sephacel. Lane I: Protein marker. Lane II: Elution profile of First peak in which we obtained HE-4 with other impurities. Lane III, IV and V: Elution profile of second, third and fourh peak respectively. (**C**) Elution profile of Sephadex G-75. The peaks were obtained as a function of X axis as elution volume in mL and Yaxis is mA at 280 nm. Buffer used for elution is 50 mM Tris-HCl pH 8.0 and 0.2 M NaCl. (**D**) 12% SDS-PAGE of the third peak of elution profile of sephadex G-75. Lane I: Protein Marker. Lane II: Elution of the third peak in non-reducing condition and Lane III: Elution profile of a third peak in reducing conditions. (**E**) Immunodetection of HE-4 in crude seminal plasma and of the third peak of elution profile of sephadex G-75. Lane I: Crude seminal plasma. Lane II: Purified protein (IIIrd peak of sephadex G-75). (**F**) The standard curve for Sephadex G-75 and lines drawn for the position of HE-4 in the standard curve.

The article "Human Epididymis Protein-4 (HE-4): A Novel Cross-Class Protease Inhibitor" was retracted in 2024. Reasons: duplicated images; overlap with earlier publications; unreliable data; concerns about the images.

**Figure 2:** Glycosylation analysis of HE-4. (**A**) PAS staining of HE-4 protein. (**B**) 12.5% SDS-PAGE of glycolsylated and unglycosylated form of HE-4 Lane I: Protein marker. Lane II: Glycosylated HE-4. Lane III: Unglycosylated HE-4.

**Table 1:** Identified Peptides of HE-4 by LC-MS/MS.

Matched Peptide	Score	Mr(expt)	Mr(calc)
K.VSCVTPNF	37	922.8927	922.4219
R.DQCQVDSQCPGQMK.C	51	1680.9627	1679.6702
R.DQCQVDSQCPGQMK.C+Oxidation (M)	51	1697.4527	1695.6651
K.CCSAGCATFCSLPNDK.E	67	1848.5127	1846.7107

WFDC-2 protein Homo sapiens (Human): Mass: 13953 Score: 123 Queries matched: 4 emPAI: 1.39.

Effect of treatment with various chemicals on solution behavior and possible aggregation pattern of native HE-4 was analyzed with dynamic light scattering (DLS). Purified HE-4 was incubated with solutions of varying pH (from acidic to alkaline) and different chemicals including various salts and reducing agents at different concentrations. The hydrodynamic radius (R_h_) of purified HE-4 (Tris-HCl buffer pH 8.0 in which protein was purified) was found to be 3.18±0.07 nm. This corresponds to approximately 46 kDa, and in complete agreement with migration of HE-4 in SDS-PAGE. Different pH had varied effect on HE-4 R_h_ values (Fig. S1A). At low pH, the R_h_ was higher which returned to native values as pH increased. Metal ions can contribute to aggregation of proteins [27] therefore we also recorded R_h_ values in the presence of various divalent metal ions and we have arranged them in decreasing order in the graph (Fig. S1A). Notably highest values were recorded in the presence of magnesium and iron salts while copper and calcium salts values were closer to the R_h_ native protein. Twenty mM ZnCl_2_ reduced the R_h_ value below native protein R_h_ value, and introduction of EDTA to the same sample in twice the molar ratio increased the Rh value, and brought it closer to the native protein. Altering pH and presence of metal ions change the solution behavior of HE-4, and may even cause the protein to adopt different conformations. As the concentration of detergents and various reducing agents increased, HE-4 R_h_ values decreased to less than that of the native protein (Fig. S1B, C and D). These DLS results, when considered with other data reported in the study support the conclusions drawn in this section.

### Sequence analysis of HE-4

Multiple sequence alignments (MSA) of HE-4 across multiple species were performed using ClustalW2 on EBI web server (Fig. 3). WFDC-2 protein sequences from different species show high similarity (Fig. 3C). Each domain consists of eight Cys residues which are fully conserved. Besides, there are other-many conserved residues a close examination of alignment reveals that these conserved residues also follow a common pattern of spacing. Comparison of the spacing between common conserved residues in each domain finds the following pattern: K(1)G(1)CP(7/11)C(3)C(2)D(2)C(4)KCC(2)GC(3/4)C(2)P, where the number in bracket represents the length of spacing. Both WAP domains of HE-4 were separately further aligned with WAP domains of other WFDC family members having anti-protease activities assigned to them (pig elafin, human elafin and human SLPI-WAP2) to gain information about function of HE-4 (Fig. 3A, B). It, reveals that in addition to C residues, K-121/72/85, P-122/73/86, G-123/74/87, P-126/77/90, M-134/85/98, N-136/87/100, P-137/88/101, P-138/89/102, N-139/90/103, D-142/95/108, K-150/103/116, G-154/107/120, G-157/110/123 and P-163/116/129 (Representations, Amino acid-position in pig elafin sequence/position in human elafin/position in human SLPI) are fully conserved, and all these may be crucial for anti-protease activity of these domains. Alignment of these domains with HE-4-WAP1 shows that out of 22 conserved residues, 3 residues including second cysteine are not conserved (C-132/83/96, M-134/85/98 and P-137/88/101), and five others are replaced by similar amino acid residues (as indicated by ‘:’ & ‘.’ in alignment). Similarly, some amino acids are not conserved, and some are substituted by similar amino acids in HE-4-WAP2. When we adjusted the optimum alignments, of HE-4-WAP1 and WAP2 domains with known antiprotease activity WAP domains, in such a way that all eight cysteine residues are perfectly conserved, and the similar pattern was observed in both alignments. Overall, six amino acid residues were found fully conserved (For HE-4-WAP1: K32, G34, P37, D52, K60, P73 and For HE-4 WAP 2: K76, G78, P81, D100, K108, P122).

The article "Human Epididymis Protein-4 (HE-4): A Novel Cross-Class Protease Inhibitor" was retracted in 2024. Reasons: duplicated images; overlap with earlier publications; unreliable data; concerns about the images.

**Figure 3:** Multiple sequence alignment of HE-4 with other WAP protein and HE-4 of different species. At the end of each line of amino acid sequence, amino acid residue numbers are given and after that % homology is written. (**A**) Sequence alignment of HE-4 WAP 1 domain with other antiproteases like elafin and WAP-2 domain of SLPI. (**B**) Sequence alignment of HE-4 WAP2 domain with other antiproteases like elafin and SLPI. (**C**) Multiple sequence alignment of HE-4 protein of human with HE-4 protein of different species.

### HE-4 is a cross-class protease inhibitor

Protease inhibition activity of HE-4 was tested according to the method of Lee and Lin [28]. Hemoglobin was used as a substrate and percentage inhibition was calculated as described in material and methods. Trypsin, chymotrysin, prostate specific antigen (PSA), proteinase K, pepsin and papain were employed for the experiment, and HE-4 showed dose-dependent inhibition of all of these proteases (Fig. 4A). The dose dependence was more for papain and pepsin and less so for other proteases. Blue native electrophoresis was performed to determine the physical complex formation of HE-4 with all the proteases (Fig. 5). All the proteases tested showed a higher molecular weight complex with HE-4 compared to HE-4 or proteases alone.

**Figure 4:** Antiprotease activity of HE-4 at different concentration and at different condition against various serine, cystine and aspartic proteases. (**A**) Percentage inhibition of various proteases like: trypsin, chymottrypsin, PSA, proteinase K, pepsin and papain by HE-4. X-axis is the HE-4 concentration in µg/ml and Y-axis is the % inhibition of respective proteases. (**B**) Effect of temperature (25°C–100°C) on the protease inhibition activity of HE-4 against trypsin. (**C**) Effect of pH (2–10) on the protease inhibition activity of HE-4 against trypsin. (**D**) Effect of different chemicals like: ZnCl_2_ SDS and β-mercaptoethanol on the protease inhibition activity of HE-4 using trypsin as model protease. EDTA was added to ZnCl_2_ pre-treated HE-4 to check whether it can rescue the decrease in activity induced by ZnCl_2._ SDS control is the % inhibition of trypsin by 5% SDS and 5% SDS point is the activity of SDS-pretreated HE-4 against trypsin. +ve control is HE-4 inhibition of trypsin without any treatment and −ve control is without HE-4, therefore 0% inhibition. (**E**) Effect of varying concentrations of EDTA on rescue of trypsin % inhibition decrease by ZnCl_2_ treatment of HE-4. (**F**) Effect of varying concentration of DTT on trypsin inhibitory activity of HE-4.

**Figure 5:** Blue native gel of HE-4 after 2 hr. incubation with different proteases. Proteases and HE-4 alone were also run to compare with the complexes formed with them. 1: Marker 45 kDa Ovalbumin, A: HE-4, B: Trypsin, C: Trypsin+HE-4, D: Chymotrypsin, E: Chymotrypsin+HE-4, F: Proteinase K, G: Proteinase K+HE-4, H: PSA, I: PSA+HE-4, J: Pepsin, K: Pepsin+HE-4, L: Papain, M: Papain+HE-4.

Effect of pH, temperature and other chemicals on HE-4 activity was tested using trypsin as a model protease. HE-4 had slightly better trypsin inhibitory activity after incubation at pH 2 and 10 while, at pH 4–6 activity was more or less similar (Fig. 4C). Effect of temperature on HE-4 inhibition of trypsin was undertaken, and activity was measured after incubation of HE-4 at different temperatures. HE-4 inhibited trypsin the most at 25°C and inhibitory activity decreased to 81% at 60°C but even after boiling at 100°C for 10 min, HE-4 retained 29% inhibition (Fig. 4B) suggesting a highly stable tertiary structure resistant to heat. This is further supported by the observation that HE-4 retained 64% inhibition of trypsin in the presence of SDS. Only 5% SDS itself showed minor inhibition of trypsin activity but much less compared to SDS-treated HE-4 (figure 4D). This suggests that SDS does not denature HE-4 significantly upto 5% concentration. Presence of β-mercaptoethanol (10% v/v) abolished the activity of HE-4 (Figure 4D). A study of effect of disulfide bond reduction on HE-4 activity against trypsin was undertaken using different concentrations of DTT. There was a significant decline in the inhibitory activity of HE-4 against trypsin (29.12%) already at 0.25 mM DTT (Figure 4F). In presence of 1 mM DTT, HE-4 completely lost its inhibitory activity (Figure 4F). This suggests that disulfide bonds based structure stabilization is essential for the protease inhibition.

The article "Human Epididymis Protein-4 (HE-4): A Novel Cross-Class Protease Inhibitor" was retracted in 2024. Reasons: duplicated images; overlap with earlier publications; unreliable data; concerns about the images.

EDTA had no effect on inhibition while 2 mM ZnCl_2_ reduced the activity to 83% and curiously, introduction of twice the molar ratio of EDTA to zinc supplemented sample restored the activity a little (Fig. 4D). Activity of HE-4 against trypsin, which decreased with ZnCl_2_ could be rescued by adding increasing concentrations of EDTA (Figure 4E).

### Interaction of HE-4 with various proteases as seen by surface plasmon resonance

HE-4 interactions with serine proteases were confirmed with surface plasmon resonance (SPR) and kinetic constants were calculated. HE-4 was immobilized on research grade CM5 chip using EDC/NHS chemistry as described in methods. Different proteases were flowed over the chip in varying concentrations, ranging from 75–300 nM. Concentration of proteases above this range was shown to reduce the signal, possibly due to “Hook effect”. Among all the proteases tested, the highest affinity (K_D_) and association constant (K_A_) was found to be for proteinase K followed by chymotrysin, PSA and then trypsin (Table 2). Trypsin had the lowest association and dissociation constants among all the proteases tested.

**Table 2:** Binding affinity of HE-4 with different proteases.

Protease	HE-4 was immobilized on CM5 chip		Proteases were immobilized on CM5 chip		HE-4 was immobilized on CM5 chip		Proteases were immobilized on CM5 chip	
	K_D_ (M)	K_A_ (M^−1^)	K_D_ (M)	K_A_ (M^−1^)	K_d_(S^−1^) [K_off_]	K_a_ (M^−1^ S^−1^) [K_on_]	K_d_(S^−1^) [K_off_]	K_a_ (M^−1^ S^−1^) [K_on_]
Proteinase K	4.65×10^−8^	2.15×10^7^	5.05×10^−8^	1.85×10^7^	9.48×10^−6^	204	10.36×10^−6^	230
Chymotrypsin	7.56×10^−8^	1.32×10^7^	7.62×10^−8^	1.17×10^7^	4.31×10^−6^	57.1	5.26×10^−6^	64.8
Trypsin	4.46×10^−4^	2.24×10^4^	5.34×10^−4^	1.96×10^4^	1.02×10^−5^	0.0229	1.62×10^−5^	0.0384
PSA	1.06×10^−5^	9.40×10^4^	1.19×10^−5^	9.23×10^4^	1.0×10^−5^	0.941	1.27×10^−5^	1.658

In separate experiments HE-4 or proteases were immobilized on CM5 chip and various proteases or HE-4 was flowed over it.

The article "Human Epididymis Protein-4 (HE-4): A Novel Cross-Class Protease Inhibitor" was retracted in 2024. Reasons: duplicated images; overlap with earlier publications; unreliable data; concerns about the images.

Converse study was also performed with SPR, where all serine proteases were on the chip and HE-4 was flowed. No significant changes were observed in binding affinity of the proteases and HE-4 (Table 2). Unfortunately, we could not determine the kinetic constants for papain and pepsin as we faced an unexpected problem of negative sensograms (Fig. 6A, B). Although, negative sensograms are not uncommon they are usually ascribed to the differences in buffer composition pre and post injection [29]. In the present study, there were no differences in the buffer compositions therefore we sought to further investigate the reason of signal dropping below baseline. For this, papain was incubated with increased concentration of HE-4 (HE-4: papain; 1∶1 to 5∶1) at pH 8.5 for 1 hr, and as a control HE-4 and papain was incubated separately for 1 hr at room temperature. Later mixtures were resolved on 14% SDS-PAGE under reducing conditions. HE-4 and papain, when incubated alone, showed band at their own molecular weight, but when they are incubated together two new bands appeared in the mixture below HE-4 band as seen in fig. 7A. In SDS-PAGE, we observed two bands that are probably the cleavage product of HE-4 by papain because with increasing concentrations of HE-4, the band at approximately 10 kDa increase in intensity while the original band of HE-4 does not increase in intensity which would be explainable by HE-4 cleavage by papain. This was confirmed with western blot which showed a low molecular weight HE-4 band lower than full length HE-4 (Figure 7C Lane 2). This explains the negative sensogram of papain (Fig. 6B) suggesting that after initial interaction with HE-4 (see the upward spike), papain cleaves and releases HE-4 from the chip bringing sensogram below baseline. In case of pepsin, we were surprised by the results as seen in fig. 7B when pepsin is incubated with HE-4(HE-4: papain; 1∶1 to 5∶1) at pH 5.0 for 1 hr it undergoes self-cleavage, as evident by the band present at approximately 20 kDa and with increasing concentration of HE-4, the decrease in intensity of pepsin (full size) band. This band at 20 kDa was definitely of pepsin as western blot using HE-4 antibodies (Figure 7C Lane 3) revealed that there was no band of HE-4 at that position. This only partially explains the sensogram of pepsin in fig. 6A and does not explain why the signal went down below the baseline unless there was also the minor cleavage of HE-4 which was not detectable in SDS-PAGE or WB because SPR would be more sensitive to even small amount of cleavage. The sensograms of other proteases were characteristic of a normal protein-protein interaction (Figure 8).

The article "Human Epididymis Protein-4 (HE-4): A Novel Cross-Class Protease Inhibitor" was retracted in 2024. Reasons: duplicated images; overlap with earlier publications; unreliable data; concerns about the images.

**Figure 6:** SPR sensograms of HE-4 interaction with papain and pepsin. Concentrations of HE-4 were fixed at 10 µM. Concentrations of papain and pepsin were 75 nM. Injection time of papain and pepsin is indicated by an arrow. (**A**) Pepsin-HE-4 interaction. (**B**) Papain-HE-4 interaction.

**Figure 7:** 14% SDS-PAGE to resolve HE-4 and pepsin, papain incubated alone or together for the same duration. (**A**) 14% SDS-PAGE (silver stained) Lane1: Molecular weight marker. Lane2: Fresh HE-4. Lane3: HE-4 after 1 hr incubation. Lane 4: Fresh papain. Lane5: papain after 1 hr incubation. Lane 6- Lane 10 papain and HE-4 in 1∶1–1∶5 (10 µg∶10 µg-10 µg∶50 µg) ratio after 1 hr incubation (in 50 mM tris-HCl buffer, pH 8.5). (**B**) 14% SDS-PAGE (silver stained) Lane1: Molecular weight marker. Lane2: Fresh HE-4 (10 µg). Lane3: HE-4 after 1 hr incubation (10 µg). Lane 4: Fresh pepsin (10 µg). Lane5: pepsin (10 µg) after 1 hr incubation. Lane 6- Lane 10 pepsin and HE-4 in 1∶1–1∶5 ratio (10 µg∶10 µg–10 µg∶50 µg) after 1 hr incubation (in 50 mM sodium acetate buffer, pH 5.0). (**C**) Immunodetection of HE-4 after incubating HE-4 alone and with pepsin and papain for the same duration. Lane1: HE-4 (10 µg) after 1 hr incubation. Lane 2: HE-4 (10 µg) after 1 hr incubation with papain (10 µg) and Lane3: HE-4 (10 µg) 1 hr incubation with pepsin (10 µg).

**Figure 8:** SPR sensograms of HE-4 interaction with serine proteases. HE-4 immobilised on CM5 chip as described in methods. Concentration of HE-4 was fixed at 10 µM. Concentrations of serine proteases (from top to bottom) were 300, 150, and 75 nM respectively. (**A**) Trypsin-HE-4 interaction. (**B**) Chymotrypsin-HE-4 interaction. (**C**) PSA- HE-4 interaction. (**D**) Proteinase K- HE-4 interaction.

## Discussion

HE-4 is upregulated in ovarian carcinoma and also expressed in a variety of lung tumors. There are several reports in the literature which suggest important functions of HE-4: over-expression in ovarian carcinoma, over-expression in prostate cancer model mice with *PTEN* inactivation, interaction with pleiotrophin (PTN) which regulates angiogenesis and is involved in tumor formation as well as the upregulation of HE-4 during the expected window of receptivity in the endometrium under the control of progesterone in primates [20], [30]–[32]. All of these evidences point towards an important role of HE-4 in human physiology but to date no study has tried to investigate the role or structure of HE-4 in normal or pathological conditions. We have developed a rapid and efficient method for purification of native HE-4 from human seminal fluid, which will help study the function and structure of HE-4.

The article "Human Epididymis Protein-4 (HE-4): A Novel Cross-Class Protease Inhibitor" was retracted in 2024. Reasons: duplicated images; overlap with earlier publications; unreliable data; concerns about the images.

### HE-4 is glycosylated and highly stable protein

HE-4 exists as a disulfide bonded trimer in human seminal fluid as inferred from SDS-PAGE in reducing and non-reducing conditions. This is not unheard of in proteins and many human and some viral proteins employ intermolecular disulfide linkages to form tertiary structure [33]–[34]. HE-4 has eight predicted disulfide bonds per monomer of protein as it is a small protein, these bonds and intermolecular disulfide linkages would be expected to give it a compact structure resistant to denaturing agents. Accordingly, it found that HE-4 is resistant to pH, heat and even SDS in protease inhibition assay taking trypsin as a model protease. Seminal fluid has a high concentration of zinc and it regulates the function of several seminal fluid proteins like PSA and sememnogelin [35].Therefore, we measured R_h_ value and activity of HE-4 in the presence of zinc and we observed lower R_h_ than that of purified native protein in Tris buffer. Introduction of EDTA in twice the molar ratio of zinc increased the R_h_ value a little bringing it closer to native HE-4. Trypsin inhibition activity of HE-4 reduced slightly in the presence of zinc (mean: 83%) while the addition of EDTA (twice the molar ratio) to the Zn supplemented HE-4 recovered the activity a little (mean: 85.6%) as shown in figure 4D. The activity lost by 2 mM ZnCl_2_ could be completely rescued by addition of increasing concentrations of EDTA (Figure 4E). At this stage evidence for mechanism of effect of zinc on activity and structure of HE-4 is inconclusive. However, this idea is being pursued further in our laboratory. Disulfide bonds play an important role in maintaining the native conformation of a protein, which in turn provide stability/resistance towards pH and temperature treatments. HE-4 contains 8 disulfide bonds. Therefore, it was of interest to evaluate the effect of DTT reduction on the trypsin inhibitory activity of HE-4. Even at .05 mM there was a significant reduction in trypsin inhibitory activity of HE-4 and at 1 mM HE-4 lost all its activity against trypsin (Figure 4F). Disulfide bond reduced HE-4 was oxidized and refolded (as described in methods) but HE-4 was unable to restore the activity and at 16 hr. time-point only 3% activity was restored. PNGase F treatment of HE-4 produced a shift of approximately 2.5 kDa which is considerable given the molecular weight of the monomer (Figure 2B). This also partly explains the observed heat and pH resistance of the protein. Asn44 has been reported to be glcyosylated in salivary HE-4 previously [36], and no other glycosylation site has been either predicted or reported. This implies that Asn44 which lies in the N-terminal WAP domain is heavily glycosylated. One previous study has reported HE-4 to be a secreted glycosylated protein of approximately 25 kDa in two ovarian carcinoma cell lines [32]. This difference with seminal fluid form of protein could be cell line specific, or it could be another isoform of the protein resulting from alternative splicing [36]. HE-4 can undergo alternative splicing to yield four different isofroms other than full length protein. Some of these isoforms has only N-terminal WAP domain and some C-terminal WAP domain while three of these isoforms own unique sequence not found in others. So this 25 kDa isoform found in ovarian cancer lines could be different from the presumably full length (based on molecular weight from SDS-PAGE) protein we have in seminal fluid, and it might even lack trimerization property, or have a different glycosylation pattern. Importance of glycosylation in functions of HE-4 (seminal fluid or other sites) requires further studies which are underway in the laboratory.

The article "Human Epididymis Protein-4 (HE-4): A Novel Cross-Class Protease Inhibitor" was retracted in 2024. Reasons: duplicated images; overlap with earlier publications; unreliable data; concerns about the images.

### HE-4 is a disulfide-bonded trimer and bioinformatic analysis alone does not correctly predict its function

A consensus sequence was obtained by aligning HE-4 sequences form different species (Fig. 3C). Though the high degree of similar conservation of residues and spacing between them points towards a similarity in functional aspects of both domains, but we cannot deny the fact that length difference between first and second cysteine residues may contribute to the different functions of these domains or the ability to covalently oligomerise, which requires inter-molecular disulfide bridges. WFDC domain of elafin and one of the two WFDC domains of SLPI is known to impart anti-proteinase activity to both of these proteins. Therefore, it is a widely held notion that all of the members of the family will have anti-proteinase activity. Sequence analysis by Bingle *et al* showed that only these two members have the same spacing between cysteines essential for protease inhibition [19]. Authors of the paper argue that no other member of the WFDC family contains the same spacing, so it is not necessary that they will have anti-proteinase activity. A separate study by Hu *et al* show that both wild type and WAP mutated KAL-1 enhanced amidolytic activity of uPA (urokinase-type plasminogen activator) [37] which are consistent with the prediction made by Bingle *et al.* This study adds a new dimension in this discussion about function of WFDC family members as we have observed antiprotease activity in HE-4. The possible reason for this discrepancy might be this spacing playing some role in inhibitory activity of SLPI and elafin. Both of these proteins are monomers while, we found HE-4 to be a disulfide bonded trimer so this rearrangement of the structure might give HE-4 unusual properties not predicted by sequence analysis. Moreover, we found that disulfide bond reduction abolishes the protease inhibition by HE-4, so we suggest that, in case of HE-4, this protease inhibition does not depend upon any of the two domains (N- and C-terminal WAP domain) alone as whole trimer seems to be necessary for the inhibition. Although one can speculate that HE-4 might be an example of inhibitors where single domains are repeated and linked together (as in ovomucoid) and this new single chain inhibitor can inhibit many different proteases [38]. The possibility of three monomers linked together by disulfide bridges point towards a compact, more rigid structure, and might resemble mechanism of ecotin in which, a homodimer is active, and both monomers provide the protease binding surface [39]. Further studies are needed to understand the mechanism of inhibition of a wide range of proteases by HE-4 which will highlight the residues crucial for inhibition; however, proximity of a variety of residues induced by trimerization might be necessary. Although we do not exclude the possibility that monomer folding pattern of HE-4 as compared to SLPI and elafin is not markedly different, so some common residues might be beneficial for protease inhibition by these proteins. Multiple sequence alignment was performed with both the WAP domains of HE-4 with WAP domains of WFDC family members having known protease inhibition activity (Fig. 3A, B). Some key amino acids which are suggested to be necessary for antiprotease activity of these domains are not conserved in HE-4, however, there is more than 70% conservation overall. More importantly, it is not always feasible to justify function of HE-4 simply on the basis of conservation of critical residues in primary sequence. Factors such as the overall structure of the domain, exposure of some specific amino acids and types of residues lining the active site may be more vital, and contribute to the activity as may be true in this study.

The article "Human Epididymis Protein-4 (HE-4): A Novel Cross-Class Protease Inhibitor" was retracted in 2024. Reasons: duplicated images; overlap with earlier publications; unreliable data; concerns about the images.

### HE-4 is cross-class protease inhibitor which is cleaved by papain and induces autolysis of pepsin in vitro

HE-4 inhibited a range of serine proteases like trypsin, chymotrypsin, PSA and proteinase K as well as cysteine proteases like papain and aspartyl proteases like pepsin. The physical complex formation of HE-4 with all these proteases was confirmed with blue native electrophoresis where complexes were migrating less compared to HE-4 or proteases alone (Figure 5). Blue native electrophoresis was chosen because some of these protease like trypsin are basic proteins therefore they do not migrate towards anode and are lost. Fig. 4A shows the protease inhibition assay results starting at 5 µg/ml concentration of HE-4 up to 50 µg/ml, and at 50 µg/ml concentration, it inhibits almost completely all the tested proteases. SLPI inhibits trypsin and chyomtrypsin with K_i_ which is not markedly different for both of these proteases [40] while HE-4 has low affinity towards trypsin and considerably higher affinity towards chymotrypsin (Table 2) as determined by SPR. This highlights different inhibition profile for HE-4 and SLPI. SLPI is thought to neutralize the excess neutrophil protease activity in upper airways. HE-4 is also expressed in sub-mucosal glands of respiratory tissues, but although SLPI and HE-4 both are found in the same tissue, the precise cells expressing both these proteins are mutually exclusive [16]. This suggests them to be under different regulatory control which point towards slightly different functions of both these proteins. HE-4 has a strong affinity towards PSA at pH 5.0 using 75–300 nm PSA (K_D_ = 1.06×10^−5^ M & K_A_ = 9.40×10^4^ M^−1^) and suggests that this protein might be involved in regulation of kallikrein activity cascades. Protein C inhibitor (PCI), α-2 macroglobulin (A2M) and α1-anti chymotrypsin (ACT) are three main inhibitors of PSA reported in human seminal fluid. Concentrations of these inhibitors in seminal fluid are low compared to PSA [41]–[43] suggesting there must be other inhibitors, which serve as main inhibitors. HE-4 seems to be one such inhibitor. PSA has been implicated in liquefaction of human seminal fluid upon ejaculation and HE-4 probably regulates the activity of PSA in semen and might protect sperm against excessive PSA activity. HE-4 inhibited proteinase K (75–300 nm) with highest affinity among the proteases tested as apparent by highest K_A_ = 2.15×10^7^ M^−1^ & K_D_ = 4.65×10^−8^ M at pH5.0 (Table 2). Proteinase K is a member of subtilisin like protease family, and it has been shown that structures of most members is conserved as a core with insertions and deletion confined to surface loops [44]. This suggests that HE-4 might be a broad spectrum inhibitor of microbial subtilisin like proteases although they need. Many pathogenic fungi utilize subtilisin-like serine proteases as their virulence factors [45]–[48] and HE-4 as a part of the host response might be conferring protection in the sites of its expression one of which is the respiratory tract, others being oral cavity and urogenital tract.

The article "Human Epididymis Protein-4 (HE-4): A Novel Cross-Class Protease Inhibitor" was retracted in 2024. Reasons: duplicated images; overlap with earlier publications; unreliable data; concerns about the images.

We could not determine the kinetics constants for HE-4 with pepsin and papain due to the negative sensogram obtained. On further investigation, we found that papain when incubated with HE-4, presents two more bands in SDS-PAGE below the molecular weight of HE-4. With increasing concentration of HE-4, the HE-4 band remains more or less same in intensity while one of the bands below it (approx 8 kDa) seems to increase in intensity and intensity of papain band also remains the same. This band of cleaved HE-4 was confirmed by western blot (Figure 7C) using HE-4 antibodies. This leads us to propose that papain cleaves HE-4 to generate low molecular weight fragments. The sensogram of papain injection over immobilized HE-4 on CM5 chip shows initial interaction and subsequent dropping of signal below baseline which is in accordance with papain cleavage of HE-4. In protease inhibition assay, HE-4 shows considerable inhibition of papain which leads us to suggest that even after cleavage, the fragment(s) of HE-4 remain(s) bound to papain inhibiting its proteolytic activity. This was confirmed with blue native electrophoresis as papain incubated with HE-4 presented only one band of high-molecular weight (Figure 5). Contrastingly, when pepsin was incubated with HE-4, it seemingly underwent self-cleavage, as evidenced by the appearance of approximately 20 kDa band which increased in intensity with increasing concentration of HE-4 with simultaneous reduction in intensity of full length pepsin band. Pepsinogen undergoes autolysis, and yield active pepsin (approximately 35 kDa) at acidic pH, while we observed a 20 kDa fragment upon incubation with HE-4. Moreover, in both the incubation experiments, we had taken control of incubating the papain and pepsin alone at appropriate pH 8.5 and 5 respectively, and these fragments of HE-4 cleavage by papain and self-cleavage of pepsin did not appear when these proteases were incubated alone. This led us to conclude that HE-4 induces the self cleavage of pepsin and papain cleaves HE-4 and the fragment of HE-4 remains active. In blue native electrophoresis we observed only one band of HE-4 (full length) when pepsin and HE-4 were incubated together (Figure 5). This suggests that pepsin cleavage also does not dissociate HE-4 from pepsin. Cysteine proteases are implicated in a variety of processes in mammalian physiology. This inhibition of papain by HE-4 fragment has greater implications for cell biology. Papain like cysteine proteases has a conserved core structure [49], and highly conserved catalytic site formed by three residues Cys25, His159, and Asn175 (papain numbering) [50]. HE-4 might inhibit other members as well, or they like papain, might be involved in cleavage of HE-4, and producing fragment, which seems to be active, although it remains speculative until further studies. IA_3_, PI-3 and equistatin, all inhibitors of cysteine proteases like papain with different specificities and targets have been isolated from different animal and microbial sources [51]. Cruzain is a papain like protease of trypanosoma cruzi, causative agent of chagas disease and its inhibitors are being looked into as possible drug development leads [52]. Structure elucidation of HE-4 and its inhibition mechanism of papain despite cleavage might help design potent inhibitors. While, on the other hand, discovery of self cleavage of pepsin when combined with protease inhibition of pepsin by HE-4 in protease inhibition assay point that HE-4 renders pepsin inactive by inducing the self-cleavage. Induced self- cleavage of a protease by a protease inhibitor has not been reported in literature previously to the best of our knowledge. This is an exceedingly curious instance, and further characterization of this phenomenon is underway in the laboratory. To confirm whether HE-4 preparation is contaminated with any endogenous protease co-purifying with HE-4, we assayed HE-4 alone with hemoglobin and BAPNA and compared to other proteases used in this study. No protease activity was found in the purified HE-4 confirming that this self-cleavage of pepsin is due to HE-4. Aspartic proteases are extremely valuable drug targets including the retroviral family and fungal aspartic proteases. Although there are structural differences between retroviral and eukaryotic pepsin-like proteases, there are similarities as well; the cleavage site loops are homologous, the Asp dyad is located in the interface region and N-terminal lobe of pepsin like enzymes are structurally similar to viral subunits [53]–[54]. HE-4 might help design better aspartic protease inhibitors in the future.

The article "Human Epididymis Protein-4 (HE-4): A Novel Cross-Class Protease Inhibitor" was retracted in 2024. Reasons: duplicated images; overlap with earlier publications; unreliable data; concerns about the images.

Finally, we can say this is the first report to establish that HE-4 is a highly stable protein which shows cross-class protease inhibition. A broad spectrum protease inhibition points towards a role in innate immunity conferring protection against microbial virulence factor of proteolytic nature. Seminal fluid HE-4 might be different from HE-4 found in other tissues like ovarian cancer cells because of alternative splicing or different glycosylation. Its ability to trimerize might not be present in all the isoforms.

## Materials and Methods

### Sample collection

Human semen samples, only normospermic (sperm count >20 million/ml, sperm motility >50%), were collected from Department of Laboratory Medicine, All India Institute of Medical Sciences (AIIMS), New Delhi, after written informed consent and the approval of the study protocol from ethics sub-committee/ethics committee of AIIMS (permit number T-03/01-04-2009). Semen samples were first subjected to liquefaction at room temperature (RT) for 30 min. Semen sample was centrifuged at 1300 g for 15 min at 4°C to separate sperm from seminal plasma. Later, for further clarification of seminal plasma supernatant was centrifuged at 7000 g for 15 min. at 4°C.

### Isolation and purification of HE-4

The supernatant, diluted with 50 mM Tris–HCl, pH7.5, containing 150 mM NaCl, was loaded on heparin–sepharose CL-6B (GE-Healthcare, Uppsala, Sweden) column. The unbound fraction was pooled separately and applied on DEAE-Sephacel column. 50 mM Tris–HCl (pH 8.0) was used as equilibration/binding buffer. After extensive washing, DEAE-sephacel bound proteins were eluted with NaCl linear gradient (0–0.5 M) in equilibration buffer. The first peak, obtained at 0.1 M NaCl, was pooled and concentrated up to 20 mg/ml by ultrafiltration (Millipore USA). Final purification of protein was achieved by size exclusion chromatography on sephadex G-75 (Sigma- Aldrich, USA) column, pre-equilibrated with 50 mM Tris–HCl (pH8.0, containing 150 mM NaCl). Fractions eluted at the flow rate of 6 ml/hr were measured at 280 nm, and pooled separately for each peak and concentrated by ultrafiltration using 3 kDa membrane cut-off. 12.5% SDS-PAGE was performed as previously described [55] to analyze approximate molecular weight and purity of the protein. Finally, gel was stained with colloidal coomassie brilliant blue (CBB).

### Kinetic analysis

#### Antiprotease activity of HE-4 against different proteases and effect of various treatments

Inhibitory activity of different serine proteases like trypsin, chymotrypsin, PSA, proteinase K and cysteine proteases like papain and aspertyl proteases like pepsin were measured with the modified method described by Lee and Lin [28]. The sample assay was as the following: 250 µl of HE-4 trimer purified from human seminal plasma was pre-incubated, at 37°C, with the same volume of proteases dissolved in 0.1 M glycine–NaOH buffer (pH 9.5) for 20 min. All the enzymes were purchased from Sigma, except PSA which was purified manually as previously described [56]. Papain and pepsin were dissolved in 50 mM ammonium acetate buffer (pH 6.5) and 50 mM sodium acetate buffer (pH 5.0) respectively. 500 µl of 1% solution of hemoglobin dissolved in the same buffer (Sigma- Aldrich, USA) was added to it, and the mixture was incubated for 40 min. The reaction was stopped by adding 2 ml of 5% trichloroacetic acid. Samples were centrifuged at 15,000 g for 10 min., and the absorbance of the supernatant was measured at 280 nm. The enzyme standard assay was as follows: 250 µl of a sample was replaced by distilled water. The chosen enzyme concentrations gave an increase of absorbance at λ°_280_ of approximately 0.005OD U/min. With purified protein (HE-4), a control assay to detect the activity of endogenous proteases was also performed: 250 µl of an enzyme solution was replaced by distilled water.

The article "Human Epididymis Protein-4 (HE-4): A Novel Cross-Class Protease Inhibitor" was retracted in 2024. Reasons: duplicated images; overlap with earlier publications; unreliable data; concerns about the images.

The percentage of inhibition was calculated as follow:Additionally, effect of temperature, pH and different chemicals on trypsin inhibition activity of HE-4 was also analyzed. For that we first incubated the 50 µg/ml of protein (HE-4) at different temperature in the range of 25°C–100°C, pH(2–10) and with different chemicals like SDS, β-mercaptoethanol, EDTA, ZnCl_2_ and ZnCl_2_+EDTA for 1 hr and the following experiments were performed as described above. In case of SDS HE-4 was incubated with 5% SDS for 2 hours before being added to trypsin and checking the activity as described above. For SDS control, inhibition of trypsin by only 5% SDS without the HE-4 was also checked as shown in fig. 4D as SDS-control. To determine the effect of zinc on HE-4 activity, HE-4 was pre-incubated with 2 mM ZnCl_2_ for 2 hr. and then activity was checked. Then in the aliquots of the same sample, different concentrations of EDTA were added and activity was checked. The effect of DTT reduction on inhibitory activity of HE-4 was examined after incubation of HE-4 with different concentrations of DTT (0.05–1.0 mM) in 25 mM NH_4_HCO_3_ for 15 min at 56°C. The reaction was terminated by adding iodoacetamide at twice the amount of each DTT concentration and the residual inhibitory activity against trypsin was determined as described above. Refolding and oxidation assay was performed as described previously [57] to check whether activity can be restored after reduction. Briefly, HE-4 was incubated at 37°C for 4 hr with 0.5 M phosphate buffer and 10 mM DTT then reaction was stopped by adding iodoacetamide (IAA) so that final concentration of IAA is 20 mM. It was dialyzed against 0.1 M KCl-HCl buffer (pH 2.0) for 3 hr. Then it was followed by dialysis against 0.01 M of the same buffer for 16 hr. at 4°C. The dialysed protein was rapidly diluted 100times with bufferA (100 mM Tris-HCl, 100 mM NaCl, 1 mM EDTA (pH 8.5), 1 mM GSH and 0.5 mM GSSG). The mixture was kept at 25°C for refolding to occur. Aliquots were withdrawn at different time intervals (0, 1, 2, 4, 8, 16 hours) and trypsin inhibitory activity was determined as described above.

The article "Human Epididymis Protein-4 (HE-4): A Novel Cross-Class Protease Inhibitor" was retracted in 2024. Reasons: duplicated images; overlap with earlier publications; unreliable data; concerns about the images.

### Blue Native gel electrophoresis

Blue Native electrophoresis was performed as described previously [58]. Briefly, all proteases were incubated with equal amount of HE-4 for 2 hours at RT. Then loading Buffer (15% glycerol, 50 mM Bistris/HCl, pH 7.0) was added to complex mixtures. Different proteases and HE-4 alone were also run in separate lane to make the comparison with complex with HE-4 and protease alone. 5–18% acrylamide gradient gel was used for separation of complexes and 50 mM tricine, 15 mM bis-tris/HCl pH 7.0 was used as cathode buffer with coomassie blue G-250 (0.002 or 0.02%). Gel was started with 0.02% coomassie G-250 in cathode buffer and after running for 1 hr it was replaced with same buffer but having 0.002% coomassie G-250 instead. 50 mM bis-tris/HCl pH 7.0 was used as anode buffer and it remained the same for the whole run. Blue native gel was performed at 4–7°C. Electrophoresis was started at 100 Volts until samples were within stacking gel. When sample reached resolving gel 15–17 mA current was applied. Gel was run for total 3–4 hr.

### Evaluation of binding potential and binding constants using SPR binding studies

The protein sensor chip was prepared by immobilization of HE-4 on a research grade CM5 chip (Biosensor AB, Uppsala, Sweden) according to the manufacturer's recommendations. SPR binding studies were performed using a BIAcore 2000TM (Biacore International, AB, and Uppsala, Sweden). 60 µl of HE-4 (30 µg/ml) in 10 mM sodium acetate buffer (pH5.0) was injected to the flow cell for 4 min at the rate of 5 µl/min and washed for 60 min at the rate of 20 µl/min. The analytes at different concentrations were injected for 4 min at a rate of 10 µl/min.

The protein samples were diluted in sodium acetate buffer pH5.0. Typically, 90 µl of different dilutions of protein were injected at a flow rate of 30 µl/min. The same buffer was passed over the sensor surface at the end of sample injection, to allow dissociation. After a 3 min dissociation phase, the sensor surface was regenerated by 30 µl of 50 mM NaOH and 1 M NaCl. The response was monitored as a function of time (sensogram) at 25°C. Binding studies were done by plotting the changes in response unit (RU) values with time (Sensograms). Kinetic constants of different proteases were calculated from the association and dissociation phases with BIA evaluation software version 3.0. Similarly converse study was also performed with SPR where all serine proteases were on the chip and HE-4 was flowed.

## Supporting Information

Figure S1 Effect of different reagents and conditions on the oligomerization of HE-4 was measured by DLS. Plot was drawn as a function of concentration of reagents and conditions as a function of X axis with hydrodynamic radii of protein on Y axis. (A) Effect of pH 2–10 empty circle) and different salt: MgCl2, FeCl2, CuCl2, CaCl2, ZnCl2 and ZnCl2+EDTA (filled circle). And (B) Effect of DTT (filled circle) and CHAPS (empty circle) in varying concentration (1%–5%). (C) Effect of SDS (filled circle) and Tween-20(empty circle) in varying concentration (2.5%–10% and 0.005%–0.05%) respectively. (D) Effect of Triton X-100(empty circle) and β-mercaptoethanol (filled circle) in varying concentration (0.1%–1.0% and the 5%–10%) respectively.
(TIF)

Supplemental Methods S1 (DOC)

The article "Human Epididymis Protein-4 (HE-4): A Novel Cross-Class Protease Inhibitor" was retracted in 2024. Reasons: duplicated images; overlap with earlier publications; unreliable data; concerns about the images.

## References

[1] Chimpanzee Sequencing and Analysis Consortium (2005) Initial sequence of the chimpanzee genome and comparison wth the human genome. Nature 437: 69–87.1613613110.1038/nature04072

[2] HurleB, SwansonW (2007) NISC Comparative Sequencing Program (2007) GreenED (2007) Green Comparative sequence analyses reveal rapid and divergent evolutionary changes of the WFDC locus in the primate lineage. Genome Res 17: 276–286.1726781010.1101/gr.6004607PMC1800918

[3] LarsenM, ResslerSJ, GerdesMJ, LuB, ByronM, et al (2000) The WFDC1 gene encoding ps20 localizes to 16q24, a region of LOHin multiple cancers. Mamm Genome 11: 767–773.1096713610.1007/s003350010135

[4] TrexlerM, BányaiL, PatthyL (2001) A human protein containing multiple types of protease-inhibitory modules. Proc Natl Acad Sci U S A 98: 3705–3709.1127438810.1073/pnas.061028398PMC31116

[5] TrexlerM, BányaiL, PatthyL (2002) Distinct expression pattern of two related human proteins containing multiple types of protease-inhibitory modules. Biol Chem 383: 223–228.1192881710.1515/BC.2002.023

[6] del CastilloI, Cohen-SalmonM, BlanchardS, LutfallaG, PetitC (1992) Structure of the X-linked Kallmann 452 syndrome gene and its homologous pseudogene on the Y chromosome. Nat Genet 2: 305–310.130328410.1038/ng1292-305

[7] TannerMM, GrenmanS, KoulA, JohannssonO, MeltzerP, et al (2000) Frequent amplification of chromosomal region 20q12–q13 in ovarian cancer. Clin Cancer Res 6: 1833–1839.10815905

[8] LarramendyML, LushnikovaT, BjörkqvistAM, WistubaII, VirmaniAK, et al (2000) Comparative genomic hybridization reveals complex genetic changes in primary breast cancer tumors and their cell lines. Cancer Genet Cytogenet 119: 132–138.1086714910.1016/s0165-4608(99)00226-5

[9] DevoogdtN, Hassanzadeh GhassabehG, ZhangJ, BrysL, De BaetselierP, et al (2003) Secretory leukocyte protease inhibitor promotes the tumorigenic and metastatic potential of cancer cells. Proc Natl Acad Sci USA 100: 5778–5782.1273271710.1073/pnas.1037154100PMC156277

The article "Human Epididymis Protein-4 (HE-4): A Novel Cross-Class Protease Inhibitor" was retracted in 2024. Reasons: duplicated images; overlap with earlier publications; unreliable data; concerns about the images.

[10] DevoogdtN, RevetsH, GhassabehGH, De BaetselierP (2004) Secretory leukocyte protease inhibitor in cancer development. Ann NY Acad Sci 1028: 380–389.1565026310.1196/annals.1322.044

[11] TianX, ShigemasaK, HirataE, GuL, UebabaY, et al (2004) Expression of human kallikrein 7 (hK7/SCCE) and its inhibitor antileukoprotease (ALP/SLPI) in uterine endocervical glands and in cervical adenocarcinomas. Oncol Rep 12: 1001–1006.15492784

[12] RobinsonPA, MarkhamAF, SchalkwijkJ, HighAS (1996) Increased elafin expression in cystic, dysplastic and neoplastic oral tissues. J Oral Pathol Med 25: 135–139.886014510.1111/j.1600-0714.1996.tb00208.x

[13] ZhangM, ZouZ, MaassN, SagerR (1995) Differential expression of elafin in human normal mammary epithelial cells and carcinomas is regulated at the transcriptional level. Cancer Res 55: 2537–2541.7780965

[14] SchalkwijkJ, WiedowO, HiroseS (1999) The trappin gene family: proteins defined by an N-terminal transglutaminase substrate domain and a C-terminal four-disulphide core. Biochem J 340: 569–577.10359639PMC1220286

[15] SallenaveJM, ShulmannJ, CrossleyJ, JordanaM, GauldieJ (1994) Regulation of secretory leukocyte proteinase inhibitor (SLPI) and elastase-specific inhibitor (ESI/elafin) in human airway epithelial cells by cytokines and neutrophilic enzymes. Am J Respir Cell Mol Biol 11: 733–741.794640110.1165/ajrcmb.11.6.7946401

[16] BingleL, CrossSS, HighAS, WallaceWA, RasslD, et al (2006) WFDC-2 (HE-4): a potential role in the innate immunity of the oral cavity and respiratory tract and the development of adenocarcinomas of the lung. Respir Res 7: 61.1660003210.1186/1465-9921-7-61PMC1459147

[17] WilliamsSE, BrownTI, RoghanianA, SallenaveJM (2006) SLPI and elafin: one glove, many fingers. Clin Sci (Lond.) 110: 21–35.1633620210.1042/CS20050115

[18] MoreauT, BarangerK, DadéS, Dallet-ChoisyS, GuyotN, et al (2008) Multifaceted roles of human elafin and secretory leukocyte proteinase inhibitor (SLPI), two serine protease inhibitors of the chelonianin family. Biochimie 90: 284–295.1796405710.1016/j.biochi.2007.09.007

[19] BingleCD, VyakarnamA (2008) Novel innate immune functions of the whey acidic protein family. Trends Immunol 29: 444–453.1867617710.1016/j.it.2008.07.001

[20] IsraeliO, Goldring-AviramA, RiensteinS, Ben-BaruchG, KorachJ, et al (2005) In silico chromosomal clustering of genes displaying altered expression patterns in ovarian cancer. Cancer Genet Cytogenet 160: 35–42.1594956810.1016/j.cancergencyto.2004.11.011

[21] KirchhoffC, HabbenI, IvellR, KrullN (1991) A major human epididymis-specific cDNA encodes a protein with sequence homology to extracellular proteinase inhibitors. Biol Reprod 45: 350–357.168618710.1095/biolreprod45.2.350

The article "Human Epididymis Protein-4 (HE-4): A Novel Cross-Class Protease Inhibitor" was retracted in 2024. Reasons: duplicated images; overlap with earlier publications; unreliable data; concerns about the images.

[22] GalganoMT, HamptonGM, FriersonHFJr (2006) Comprehensive analysis of HE-4 expression in normal and malignant human tissues. Mod Pathol 19: 847–53.1660737210.1038/modpathol.3800612

[23] SchanerME, RossDT, CiaravinoG, SorlieT, TroyanskayaO, et al (2003) Gene expression patterns in ovarian carcinomas. Mol Biol Cell 14: 4376–4386.1296042710.1091/mbc.E03-05-0279PMC266758

[24] HellstromI, RaycraftJ, Hayden-LedbetterM, LedbetterJA, SchummerM, et al (2003) The HE-4 (WFDC-2) protein is a biomarker for ovarian carcinoma. Cancer Res 63: 3695–3700.12839961

[25] DrapkinR, von HorstenHH, LinY, MokSC, CrumCP, et al (2005) Human epididymis protein 4 (HE-4) is a secreted glycoprotein that is overexpressed by serous and endometrioid ovarian carcinomas. Cancer Res 65: 2162–2169.1578162710.1158/0008-5472.CAN-04-3924

[26] RamachandranP, BoontheungP, XieY, SondejM, WongDT, et al (2006) Identification of N-linked glycoproteins in human saliva by glycoprotein capture and mass spectrometry. J Proteome Res 5: 1493–1503.1674000210.1021/pr050492k

[27] JinL, WuWH, LiQY, ZhaoYF, LiYM (2011) Copper inducing Aβ42 rather than Aβ40 nanoscale oligomer formation is the key process for Aβ neurotoxicity. Nanoscale 3: 4746–4751.2195255710.1039/c1nr11029b

[28] LeeTM, LinYH (1995) Trypsin inhibitor and trypsin-like protease activity in air- or submergence-grown rice (Oryza sativa L.) coleoptiles. Plant Science 106: 43–54.

[29] ChouCL, Sadegh-NasseriS (2000) HLA-DM Recognizes the Flexible Conformation of Major Histocompatibility Complex Class II. J Exp Med 192: 1697–1706.1112076710.1084/jem.192.12.1697PMC2213500

[30] KorstenH, Ziel-van der MadeA, MaX, van der KwastT, TrapmanJ, et al (2009) Accumulating progenitor cells in the luminal epithelial cell layer are candidate tumor initiating cells in a Pten knockout mouse prostate cancer model. PLoS One 4: e5662.1946189310.1371/journal.pone.0005662PMC2680948

[31] StelzlU, WormU, LalowskiM, HaenigC, BrembeckFH, et al (2005) A human protein-protein interaction network: a resource for annotating the proteome. Cell 122: 957–968.1616907010.1016/j.cell.2005.08.029

[32] AceCI, OkuliczWC (2004) Microarray profiling of progesterone-regulated endometrial genes during the rhesus monkey secretory phase. Reprod Biol Endocrinol 2: 54.1523983810.1186/1477-7827-2-54PMC471571

[33] Perez-VilarJ, HillRL (1997) Norrie disease protein (norrin) forms disulfide-linked oligomers associated with the extracellular matrix. J Biol Chem 272: 33410–33415.940713610.1074/jbc.272.52.33410

[34] LiPP, NakanishiA, ClarkSW, KasamatsuH (2002) Formation of transitory intrachain and interchain disulfide bonds accompanies the folding and oligomerization of simian virus 40 Vp1 in the cytoplasm. Proc Natl Acad Sci U S A 99: 1353–1358.1180530410.1073/pnas.032668699PMC122194

The article "Human Epididymis Protein-4 (HE-4): A Novel Cross-Class Protease Inhibitor" was retracted in 2024. Reasons: duplicated images; overlap with earlier publications; unreliable data; concerns about the images.

[35] De LamirandeE (2007) Semenogelin, the main protein of the human semen coagulum, regulates sperm function. Semin Thromb Hemost 33: 60–68.1725319110.1055/s-2006-958463

[36] BingleL, SingletonV, BingleCD (2002) The putative ovarian tumour marker gene HE-4 (WFDC-2), is expressed in normal tissues and undergoes complex alternative splicing to yield multiple protein isoforms. Oncogene 21: 2768–27673.1196555010.1038/sj.onc.1205363

[37] HuY, González-MartínezD, KimSH, BoulouxPM (2004) Cross-talk of anosmin-1, the protein implicated in X-linked Kallmann's syndrome, with heparan sulphate and urokinase-type plasminogen activator. Biochem J 384: 495–505.1532430210.1042/BJ20041078PMC1134135

[38] TokuishiK, YamashitaS, OhboK, KawaharaK (2012) Splice variant HE-4-V3 expression is associated with favorable prognosis in pulmonary adenocarcinoma. Tumour Biol 33: 103–109.2201592910.1007/s13277-011-0252-8

[39] ArdeltW, LaskowskiMJr (1985) Turkey ovomucoid third domain inhibits eight different serine proteinases of varied specificity on the same …Leu18-Glu19… reactive site. Biochemistry 24: 5313–5320.390770010.1021/bi00341a007

[40] EggersCT, WangSX, FletterickRJ, CraikCS (2001) The role of ecotin dimerization in protease inhibition. J Mol Biol 308: 975–991.1135258610.1006/jmbi.2001.4754

[41] EisenbergSP, HaleKK, HeimdalP, ThompsonRC (1990) Location of the protease-inhibitory region of secretory leukocyte protease inhibitor. J Biol Chem 265: 7976–7981.2110563

[42] SchillWB (1976) Quantitative determination of high molecular weight serum proteinase inhibitors in human semen. Andrologia 8: 359–364.108753810.1111/j.1439-0272.1976.tb01671.x

[43] BirkenmeierG, UsbeckE, SchäferA, OttoA, GlanderHJ (1998) Prostate-specific antigen triggers transformation of seminal alpha2-macroglobulin (alpha2-M) and its binding to alpha2-macroglobulin receptor/low-density lipoprotein receptor-related protein (alpha2-M-R/LRP) on human spermatozoa. Prostate 36: 219–225.971902110.1002/(sici)1097-0045(19980901)36:4<219::aid-pros2>3.0.co;2-a

[44] AhlgrenG, RannevikG, LiljaH (1995) Impaired secretory function of the prostate in men with oligo-asthenozoospermia. J Androl 16: 491–498.8867597

[45] SiezenRJ, de VosWM, LeunissenJA, DijkstraBW (1991) Homology modelling and protein engineering strategy of subtilases, the family of subtilisin-like serine proteinases. Protein Eng Oct 4: 719–737.10.1093/protein/4.7.7191798697

[46] HuangX, ZhaoN, ZhangK (2004) Extracellular enzymes serving as virulence factors in nematophagous fungi involved in infection of the host. Res Microbiol 155: 811–816.1556727410.1016/j.resmic.2004.07.003

The article "Human Epididymis Protein-4 (HE-4): A Novel Cross-Class Protease Inhibitor" was retracted in 2024. Reasons: duplicated images; overlap with earlier publications; unreliable data; concerns about the images.

[47] St LegerRJ (1995) The role of cuticle-degrading proteases in fungal pathogenesis of insects. Can J Bot 73: 1119–1125.

[48] SreedharL, KobayashiDY, BuntingTE, HillmanBI, BelangerFC (1999) Fungal proteinase expression in the interaction of the plant pathogen Magnaporthe poae with its host. Gene 235: 121–129.1041534010.1016/s0378-1119(99)00201-2

[49] BryantMK, SchardlCL, HesseU, ScottB (2009) Evolution of a subtilisin-like protease gene family in the grass endophytic fungus Epichloë festucae. BMC Evol Biol 9: 168.1961510110.1186/1471-2148-9-168PMC2717940

[50] DickinsonDP (2002) Cysteine peptidases of mammals: their biological roles and potential effects in the oral cavity and other tissues in health and disease. Crit Rev Oral Biol Med 13: 238–275.1209046410.1177/154411130201300304

[51] LecailleF, KaletaJ, BrömmeD (2002) Human and parasitic papain-like cysteine proteases: their role in physiology and pathology and recent developments in inhibitor design. Chem Rev 102: 4459–4488.1247519710.1021/cr0101656

[52] SajidM, RobertsonSA, BrinenLS, McKerrowJH (2011) Cruzain: the path from target validation to the clinic. Adv Exp Med Biol 712: 100–115.2166066110.1007/978-1-4419-8414-2_7

[53] TangJ, JamesMN, HsuIN, JenkinsJA, BlundellTL (1978) Structural evidence for gene duplication in the evolution of the acid proteases. Nature 271: 618–621.2417910.1038/271618a0

[54] BlundellTL, SrinivasanN (1996) Symmetry, stability, and dynamics of multidomain and multicomponent protein systems. Proc Natl Acad Sci USA 93: 14243–14248.896203310.1073/pnas.93.25.14243PMC34468

[55] LaemmliUK, MölbertE, ShoweM, KellenbergerE (1970) Form-determining function of genes required for the assembly of the head of bacteriophage T4. J Mol Biol 49: 99–113.545052010.1016/0022-2836(70)90379-7

[56] HassanMI, KumarV, KashavT, AlamN, SinghTP, et al (2007) Proteomic approach for purification of seminal plasma proteins involved in tumor proliferation. J Sep Sci 30: 1979–1988.1763836210.1002/jssc.200700028

[57] PandhareJ, DeshpndeV (2004) Both chaperone and isomerase functions of protein disulfide isomerase are essential for acceleration of the oxidative refolding and reactivation of dimeric alkaline protease inhibitor. Protein Sci 13: 2493–501.1529510810.1110/ps.03552004PMC2280025

[58] SchäggerH, CramerWA, von JagowG (1994) Analysis of molecular masses and oligomeric states of protein complexes by bluenative electrophoresis and isolation of membrane protein complexes by two-dimensional native electrophoresis. Anal Biochem 217: 220–30.820375010.1006/abio.1994.1112

